The article "Hydrogen sulfide protects H9c2 cardiomyoblasts against H2O2-induced apoptosis" was published in 2019. Journal: Braz J Med Biol Res.

# Hydrogen sulfide protects H9c2 cardiomyoblasts against H_2_O_2_-induced apoptosis

**DOI:** 10.1590/1414-431X20187626

**Published:** 2019-04-15

**Authors:** You En Zhang, Guang Qing Huang, Bing Wu, Xin Duo Lin, Wen Zi Yang, Zun Yu Ke, Jie Liu

**Affiliations:** 1 Department of Cardiology, Institute of Clinical Medicine, Renmin Hospital, Hubei University of Medicine, Shiyan, China; 2 Department of Intensive Care Unit, Renmin Hospital, Hubei University of Medicine, Shiyan, China; 3 Department of Neurology, Renmin Hospital, Hubei University of Medicine, Shiyan, China

**Keywords:** Reactive oxygen species, ROS, Hydrogen sulfide, H_2_O_2_-induced apoptosis, Cardiomyocytes

## Abstract

Reactive oxygen species (ROS) are highly reactive chemical species that may cause irreversible tissue damage, and play a critical role in cardiovascular diseases. Hydrogen sulfide (H_2_S) is a gasotransmitter that acts as a ROS scavenger with cardio-protective effects. In this study, we investigated the cytoprotective effect of H_2_S against H_2_O_2_-induced apoptosis in cardiomyocytes. H9c2 rat cardiomyoblasts were treated with H_2_S (100 μM) 24 h before challenging with H_2_O_2_ (100 μM). Apoptosis was then assessed by annexin V and PI, and mitochondrial membrane potential was measured using a fluorescent probe, JC-1. Our results revealed that H_2_S improved cell viability, reduced the apoptotic rate, and preserved mitochondrial membrane potential. An increased Bcl-2 to Bax ratio was also seen in myocytes treated with H_2_S after H_2_O_2_-induced stress. Our findings indicated a therapeutic potential for H_2_S in preventing myocyte death following ischemia/reperfusion.

## Introduction

Reactive oxygen species (ROS) are highly reactive chemical species from cellular metabolism involving oxygen consumption (1). In normal tissues, approximately 5% of the consumed oxygen molecules are transformed into ROS (2). These ROS can initiate chain reactions in tissues, leading to irreversible damage in proteins, lipids, and nucleic acids (1). ROS play an essential role in regulating cell activities, such as gene expression, cell growth, and cell death (3). ROS can be detoxified by endogenous enzymes or free radical scavengers. However, the imbalance between antioxidants and oxidants leads to overproduction of ROS. This effect is associated with many multifactorial diseases, such as cardiovascular disorders (4,5). Global ischemia and reperfusion have been associated with the upregulation of ROS in cardiomyocytes (e.g., hydrogen peroxide [H_2_O_2_]), resulting in oxidative stress injuries (6). H_2_O_2_ may cause apoptosis in cardiomyocytes by activating the intrinsic apoptotic pathways. Therefore, H_2_O_2_ is often utilized to establish an *in vitro* model for ischemia and subsequent reperfusion (I/R) injury (4,5).

The article "Hydrogen sulfide protects H9c2 cardiomyoblasts against H2O2-induced apoptosis" was published in 2019. Journal: Braz J Med Biol Res.

Hydrogen sulfide (H_2_S) is predominantly synthesized from L-cysteine via cystathionine γ-lyase in the heart and vasculature. H_2_S has drawn great scientific interest regarding myocardial protection. H_2_S possesses almost all the beneficial cardiovascular effects similar to another well-characterized gasotransmitter, nitric oxide (NO) (7). Moreover, H_2_S acts as a ROS scavenger without producing deleterious ROS, which is typically seen in NO. H_2_S is rapidly emerging as a novel lipophilic cytoprotective signaling molecule with potent antioxidant, anti-inflammatory, and anti-apoptotic features (8,9). Our previous *in vivo* study revealed that the exogenous H_2_S donor, sodium hydrosulfide (NaHS), has potent anti-inflammatory effects in the heart damaged by acute myocardial infarction, which may be partially due to the limited CD11b^+^Gr-1^+^ myeloid cells (10).

Although we have discovered the physiological and cardioprotective effects of H_2_S, the signaling mechanisms that mediate these effects have not been thoroughly evaluated. This study aimed to elucidate the mechanisms by which H_2_S prevents apoptosis of cardiomyocytes. In particular, we studied the mitochondrial pathway in response to H_2_O_2_-induced oxidative stress using an *in vitro* model that mimicked ischemia-reperfusion injuries.

## Material and Methods

### H_2_S donor

H_2_S was administered in the form of sodium hydrosulfide (NaHS) (Sigma-Aldrich, Cat. No.161527, USA). NaHS was freshly prepared in normal saline (0.9%) to the desired concentration before administration.

### Cell culture

H9c2 cells (rat cardiomyoblasts) were obtained from the Cell Bank of the Chinese Academy of Sciences (China), and grown at a density of 10^5^ cells/cm^2^ as a monolayer. H9c2 cells were cultured in Dulbecco's modified Eagle medium (GIBCO, Cat. No. 11960-077, USA) supplemented with 10% v/v fetal bovine serum, 2 mM glutamine, 1% nonessential amino acids, 100 IU penicillin, and 100 μg/mL streptomycin under an atmosphere of 5% CO_2_ saturated with water vapor at 37°C. The medium was replaced by fresh medium every two days. Subculture was done when the plates were more than 90% confluency.

### Hydrogen peroxide treatment

To induce oxidative stress in H9c2 cells, the cells were cultured in serum-free medium containing 100 μM H_2_O_2_ for 24 h with or without a 30 min pre-treatment of 100 μM NaHS. H_2_O_2_ and NaHS were freshly prepared before each experiment. Control groups were treated with both H_2_O_2_ and NaHS simultaneously.

### Apoptosis assay

An annexin V apoptosis detection kit (BD Biosciences, Cat. No. 556547, USA) was utilized to measure apoptosis of H2c9 cells following the manufacturer's instruction. After treatments, cells were washed twice with cold PBS, trypsinized, and then resuspended in the binding buffer at a concentration of 1×10^6^ cells/mL. A 100 μL-aliquot of the cell suspension (1×10^5^ cells) was then incubated with fluorescein isothiocyanate (FITC)-annexin V and propidium iodide for 15 min at room temperature in the dark. Apoptotic rate was analyzed using flow cytometry within 1 h.

The article "Hydrogen sulfide protects H9c2 cardiomyoblasts against H2O2-induced apoptosis" was published in 2019. Journal: Braz J Med Biol Res.

### Measurement of ROS production

The presence of intracellular ROS was detected using dihydroethidium (DHE, Sigma, Cat. No. D7008, USA), a sensitive fluorescent dye. According to the manufacturer's instructions, sub-confluent cells were pre-treated with or without 100 μM NaHS for 30 min, and then further incubated with 100 μM H_2_O_2_ for 24 h. Cells were then washed with PBS and incubated with 5 μM DHE at 37°C for 30 min. Fluorescence was captured with a fluorescent microscope, and the signal intensity was reported as a percentage of the control group.

### Measurement of mitochondrial membrane potential (&b_psgr;_m_)

Changes in the ψ_m_ were detected using a mitochondria-specific cationic dye, JC-1 (Life Technologies, Cat. No. T3168, USA). JC-1 is a lipophilic cation that can selectively enter into mitochondria. H9c2 cells with or without H_2_O_2_ treatment were incubated with 10 μg/mL JC-1 at 37°C in the dark for 10 min. The loading solution was then replaced with fresh medium, and the fluorescent signal was captured and analyzed using the fluorescence microscopy. Red emission indicates membrane potential-dependent JC-1 aggregates in mitochondria. Green fluorescence reflects the monomeric form of JC-1 appearing in the cytoplasm after mitochondrial membrane depolarization. Consequently, mitochondrial depolarization is indicated by a decrease in the red/green fluorescence intensity ratio.

### Western blot analysis

Western blot analysis was performed as previously described (11). Total protein lysates were collected for the standard immunoblot analysis. Protein concentrations were determined by a BCA protein assay. Aliquots of protein lysates (30 μg/lane) were loaded into sodium dodecyl sulfide-polyacrylamide gels (SDS-PAGE) and transferred to the PVDF membrane. The membrane was blocked and incubated with Bcl-2, Bax, and activated-caspase 3 p17 primary antibodies overnight at 4°C. Bcl-2 and Bax antibodies were purchased from Cell Signaling Technology (USA) (Bcl-2 Cat. No. 3498; Bax Cat. No. 14796), and activated-caspase 3 p17 antibody was from Bioworld (Cat. No. BS7004, USA). Blots were washed with TBST (Sigma-Aldrich), followed by incubation with corresponding horseradish peroxidase-conjugated secondary antibodies (Jackson Laboratory, USA). Lastly, the blots were visualized with enhanced chemiluminescence and were quantified by densitometry.

The article "Hydrogen sulfide protects H9c2 cardiomyoblasts against H2O2-induced apoptosis" was published in 2019. Journal: Braz J Med Biol Res.

### Statistical analysis

Data are reported as means±SE. Different groups were compared using one-way analysis of variance (ANOVA) followed by the Student-Newman-Keuls *post hoc* test. Comparison between two groups was assessed by *t*-test. P<0.05 was considered statistically significant.

## Results

### H_2_S reduced H_2_O_2_-induced apoptosis

To determine whether H_2_S affected H_2_O_2_-induced apoptosis in H2c9 cells, we performed annexin V & PI assays. Flow cytometry was then utilized to evaluate the apoptotic rate (Figure 1A). Compared to the control group, H_2_O_2_ significantly induced cell apoptosis, but the presence of H_2_S rescued H_2_O_2_ cytotoxicity, and increased cell viability (Figure 1B).

**Figure 1.** Hydrogen sulfide (H_2_S) reduced H_2_O_2_-induced H9c2 apoptosis. **A**, Cell death analysis of treated cells was performed by flow cytometry with annexin V/PI double staining. Representative quantitative analysis is shown in **B**. Data are reported as means±SE (n=6). *P<0.05, **P<0.01 *vs* control; ^#^P<0.05, ^##^P<0.01 *vs* NaHS; ^&^p<0.01 *vs* H_2_O_2_ (ANOVA followed by Student-Newman-Keuls *post hoc* test).

### H_2_S protected H9c2 cells from oxidative stress

Oxidative stress leads to detrimental changes in the cell signaling process. To determine whether H_2_S has any effect on ROS activity under oxidative stress, we examined total ROS levels using DHE. Compared to the control group, H9c2 cells with H_2_O_2_ treatment showed an enhancement of fluorescence intensity by approximately six-fold. However, pre-treatment with H_2_S demonstrated a significant rescue effect (50.2% reduction of the fluorescence intensity) (Figure 2).

**Figure 2.** Hydrogen sulfide (H_2_S) protected H9c2 cells against H_2_O_2_-induced oxidative stress (**A**). Intracellular superoxide anion production was detected with dihydroethidium and observed by fluorescent microscopy (**B**). The fluorescent signal was measured and quantified. Data are reported as means±SE (n=6). *P<0.01 *vs* control; ^#^P<0.01 *vs* NaHS; ^&^P<0.01 *vs* H_2_O_2_ (ANOVA followed by Student-Newman-Keuls *post hoc* test). ROS: reactive oxygen species.

### H_2_S prevented the loss of mitochondrial membrane potential (&b_psgr;_m_)

Mitochondrial function is highly sensitive to oxidative damages. In this study, we applied the fluorescent dye JC-1 to investigate whether H_2_S protected the physical functions of mitochondria from H_2_O_2-_induced cell stress in the cell model. In the control group, H9c2 cells exhibited numerous brightly stained mitochondria that emitted orange fluorescence (Figure 3A). After treating with H_2_O_2_ for 24 h, H9c2 cells demonstrated fewer and less stained mitochondria (Figure 3B). H_2_S pre-treatment, on the other hand, prevented H_2_O_2_-induced loss of mitochondrial membrane potential.

The article "Hydrogen sulfide protects H9c2 cardiomyoblasts against H2O2-induced apoptosis" was published in 2019. Journal: Braz J Med Biol Res.

**Figure 3.** Hydrogen sulfide (H_2_S) prevented the loss of mitochondrial membrane potential (ψ_m_) (**A**). The ψ_m_ loss was determined by the lipophilic cationic probe JC-1. Red signal indicates JC-1 in mitochondria and green signal indicates cytosolic JC-1. Magnification ×400; bar: 50 μm. **B**, Quantitative analysis of membrane potential. Data are reported as means±SE (n=6). *P<0.01 *vs* control; ^#^P<0.01 *vs* NaHS; ^&^P<0.05 *vs* H_2_O_2_ (ANOVA followed by the Student-Newman-Keuls *post hoc* test).

### H_2_S regulated the expression of apoptosis-related proteins

Compared to the expression levels of H_2_O_2_-treated H9c2 cells, the protein expression level of Bax was significantly reduced, while Bcl-2 expression was increased in the NaHS-treated cells (Figure 4A). Consequently, compared with the H_2_O_2_ group, the ratio of Bcl-2 to Bax was higher in the NaHS + H_2_O_2_ group (Figure 4B-D). The expression level of activated caspase 3, another apoptotic marker, was also examined (Figure 4E). The results suggested that H_2_O_2_ enhanced apoptosis in H9c2 cells, while the NaHS treatments decreased H_2_O_2_-induced apoptosis.

**Figure 4.** Hydrogen sulfide (H_2_S) regulated the expression of apoptosis-related proteins. **A**, Representative immunoblots showing the expression of Bax, Bcl-2, and activated caspase 3 p17 in the H9c2 cells. Bax (**B**) and Bcl-2 (**C**) expression normalized to GAPDH (n=6). **D**, Densitometric analysis of the ratio of Bcl-2 to Bax. **E**, Activated caspase 3 p17 expression normalized to GAPDH. Data are reported as means±SE (n=6) (ANOVA followed by Student-Newman-Keuls *post hoc* test). NS: not significant.

## Discussion

As a gaseous signaling molecule, H_2_S can freely diffuse across cell membranes and activate various cellular targets. This distinct feature makes H_2_S an attractive pharmacological agent to treat cardiovascular diseases. Previous studies have demonstrated a compelling cardioprotective effect of H_2_S in rat and mouse models (12 [Bibr B13]–14). We have shown that H_2_S pre-treatment efficiently protected human ventricular fibroblasts from H_2_O_2_-induced endoplasmic reticulum (ER) stress and prevented the activation of caspase cascade (15). In the current study, we showed that H_2_S protected H9c2 cardioblasts from H_2_O_2_-induced oxidative stress. H_2_S regulated the cell cycle, decreased apoptotic cells, and preserved mitochondrial membrane potential ψm that is essential for ATP production and homeostasis. H_2_S also upregulated Bcl-2/Bax ratio, suggesting its critical role in the anti-apoptotic mechanisms. Both studies indicated the holistic role of H_2_S in protecting the cardiovascular system.

The article "Hydrogen sulfide protects H9c2 cardiomyoblasts against H2O2-induced apoptosis" was published in 2019. Journal: Braz J Med Biol Res.

Oxidative stress is the imbalance between ROS production and detoxification. This imbalance impairs the capacity to repair the damages caused by reactive intermediates. Moreover, imbalance in oxidative states may lead to the generation of peroxides and free radicals, which in turn damage proteins, lipids, and DNA (1). Oxidative damage from H_2_O_2_ contributes to heart failure and tissue damages (16). The H_2_O_2_ molecule plays an essential role in the progression of oxidative stress and cardiac pathologies (17,18). In addition, excessive ROS damages mitochondria, opens its permeability transition pore (PTP), and thus induces mitochondrial permeability transition. These alterations cause mitochondrial depolarization and outer membrane rupture, leading to cell apoptosis or death (19,20). Apoptosis that occurs in the clinical setting (*e.g.*, open-heart surgery under cardiopulmonary bypass) is induced by various conditions and agents, including ROS, NO, calcium, and pressure overload, mechanical stress, tumor necrosis factor, and angiotensin II. Apoptosis has also been shown to play a pivotal role in the pathogenesis of ischemia/reperfusion (21).

Endogenous gaseous signaling mediators, such as H_2_S, are formed in mammalian cells and tissues. H_2_S may easily react with certain compounds, especially with reactive oxygen and nitrogen species, such as superoxide radical anion (O_2_-), H_2_O_2_, peroxynitrite (ONOO-), and hypochlorite (ClO-) (22 [Bibr B23]–24). In the current study, we demonstrated that H_2_O_2_ induced ROS production and decreased mitochondrial membrane potential, suggesting an impairment of mitochondrial functions. H_2_S treatment, however, attenuated the ROS production, restored mitochondrial membrane potential, and decreased cardiomyocyte apoptosis. H_2_S may protect mitochondrial function via multiple pathways, such as activating AMPK in cardiomyocytes (25).

Previous studies showed that Bcl-2 family is upregulated during the opening of PTP (19,20). PEP-1-CAT, a fusion protein of anti-microbial peptide and antioxidant enzyme, protects cardiomyocyte from hypoxia/reoxygenation-induced injuries. PEP-1-CAT blocks Bcl-2/Bax/mitochondrial apoptotic pathway by inhibiting p38 MAPK while activating the PI3K/Akt and Erk1/2 signaling pathways (26). Here, we also found H_2_S regulated the Bcl-2/Bax/caspase-3 signaling pathway in the rat cardiomyoblasts. The functions of Bcl-2 (anti-apoptosis) and Bax (pro-apoptosis) proteins are in opposition of the apoptotic pathway. When the apoptotic signal is present, caspase 3 (32 kD) will be cleaved and present as an active form (17 kD) to induce cell apoptosis (27). In our study, H_2_O_2_ treatment led to a shift in favor of the pro-apoptotic protein, Bax, as well as upregulated the downstream effector, caspase 3. On the other hand, H_2_S rescued this apoptotic event and downregulated the level of caspase 3, demonstrating a cytoprotective effect in the rat cardiomyoblasts.

The article "Hydrogen sulfide protects H9c2 cardiomyoblasts against H2O2-induced apoptosis" was published in 2019. Journal: Braz J Med Biol Res.

In conclusion, we demonstrated that NaHS has potent anti-apoptotic effects in cardiomyoblasts with H_2_O_2_-induced injuries. The anti-apoptotic function may be partially due to blocking ROS production in mitochondria, maintaining mitochondrial membrane integrity, and inhibiting activation of the Bcl-2/Bax apoptotic pathway. The current study suggested that H_2_S may serve as an effective therapeutic option for treating ischemia-reperfusion injuries.
